# Self-Psychological Control and Creativity of Music Creation in Multimusic Environment

**DOI:** 10.1155/2022/7849909

**Published:** 2022-07-08

**Authors:** Caihong Xu

**Affiliations:** The Department of Music, Yuncheng University, Yuncheng, Shanxi, China

## Abstract

This study aimed to solve the difficulties in the research of self-psychology, three executive controls, and creativity in multimusic environment. In today's teaching and performance, the study of piano adaptation has practical significance in broadening artistic vision, improving performance technology, and training symphonic music thinking. A research method of self-psychological three executive controls and creativity generation for creation in multimusic environment is proposed. A computer composition algorithm is based on the hidden Markov model and interactive genetic algorithm. By integrating melody elements and rhythm into the traditional Markov model with only notes or rhythm as the unit, a new hidden Markov music prediction model is established, and the interactive genetic algorithm is used to optimize the music segments. Simulation results show that the algorithm can use a small dataset to quickly create music clips with certain melody logic and in line with users' personality. It is proved that the method based on the hidden Markov model and interactive genetic algorithm can meet the research needs of self-psychological three execution control and creativity generation in multimusic environment.

## 1. Introduction

The environment in which music is created is an important determinant and the diversity of environments allows for a wide range of possibilities. One of the most important influences is the natural environment, and through self-psychological control, it can help save carbon emissions in the process of creating music, while creating music that conveys a desire for the beauty of the natural environment and causes more people to be aware of the need to protect it.

In the vast number of piano music works, there are always some differences in the value judgment of adapted music. The so-called piano adaptation is adapted from other forms of music works and transformed into piano works through keyboard music thinking. In the history of music, the number of piano adaptations is extremely large. Whether out of artistic interest or practical needs, this music form has continued since the birth of the piano, especially in the romantic period. On the other hand, because the adaptation cannot be completely separated from the influence of the original and there are some rough adaptation works, the creation form of piano adaptation has objections in the evaluation of artistic independence and artistic quality. However, from the perspective of the development of macromusic history and the current situation of piano performance and teaching, piano adaptation still has irreplaceable significance. This study focuses on the excellent piano adaptation in the history of music, discusses its historical factors and artistic characteristics, and extends it to the current development context of piano music in China, trying to further clarify the practical significance of piano adaptation in performance and teaching [1]. However, in teaching of piano performance, the induction of theory, technology, and practice is also very important, as shown in Figure 1.

In the context of international culture, in order to improve the quality and innovation capacity of all cultures, it is necessary to apply the concept of multicultural education, music, and support music education in our country. The significance of this concept is as follows: (1) meet the current needs of economic globalization and cultural diversity. At present, people have entered the information age. There are frequent exchanges and collisions between various cultures. Cultural diversity has become a key consensus in the world. Based on this, actively promoting the progress of the multicultural education model is to comply with the pace of the progress of the times. At the same time, carrying out multicultural education in college education activities can promote students to look at the music culture of each region and each nation with a broader vision, promote mutual reference and learning among all ethnic groups to a great extent, and strengthen cooperation and exchange among all ethnic groups [2]. (2) It is conducive to improving national quality and promoting the construction of a civilized and powerful country and a harmonious society. Music education is an important form of cultural education, which can improve the comprehensive quality and cultural soft power of the people. By further carrying out multicultural music education, it can comprehensively promote the process of social harmonious development composed of people from various cultural backgrounds, which is conducive to the revitalization of the country and the nation. (3) It is conducive to the reform and innovation of music education, the active implementation of multicultural music education, and the use and excavation of China's long-standing and profound national music culture to a great extent, which can break the pattern of Western music Monism and make China's music education more diversified in content and form [3], as shown in Figure 2.

## 2. Literature Review

Multicultural music education is as much a concept as multicultural education. Many experts, scholars, and researchers explain this based on their research. Lim, the founder of the concept of music education, understands the changing nature of diversity in a variety of music genres around the world. The difference in music is due to the presence of music in the culture. Cultural differences determine the diversity of music, and the study of music depends on the diversity of music, which inevitably reflects the diversity of characteristics [4]. The multicultural music education has been recognized as a form of music science and music planning. He believes this is a model of multicultural music education. Zheng, vice president of the China' World Music Association, defines that the concept of multicultural music education is a multicultural, multicultural culture that reflects the history of people and music education and the development of one another. Therefore, music education should dismantle Western music, especially European music, and embrace all the world music and culture. First of all, we must acknowledge and adhere to the culture of different cultures of all races and use the music and culture exchange and discussion of the countries [5].

In short, multicultural music education, as a multicultural education sector, seeks to promote the richness and diversity of music education and to develop diversity and a round to equal music education for all cultures around the world, the success of the heterogeneity of music culture. Specialized study topics include Western music, modern star music, Western music, and non-Western music. It is a standard pan-cultural music education that includes all aspects of music culture from ancient times to the present. The goal is to expand students' esthetic perceptions by learning a variety of music, increasing understanding and respect for different cultures, helping students set up music standards, and make students face more of the challenges of globalization in the future.

In music creation, adaptation has existed since ancient times. According to the literature, organ adaptation has appeared since the 14th century, and the adaptation phenomenon in the composer's creation is also very common in the Baroque period and the classical period. However, different from the romantic period, the early keyboard music adaptation is more out of the composer's creative will. It is a type of music genre, and it also realizes the reference and learning of others' creations through adaptation. Bianco has made achievements in the adaptation of his own works and the creation of others, which not only shows his artistic interest but also shows the artistic commonality of Baroque music for future generations [6]. Kengerli-Najafova, the early seven piano concertos were all adapted from the creations of others. For example, the three piano concertos numbered k.107 came from his three piano sonatas [7]. It should be said that Mozart benefited a lot from this kind of adaptation in his early artistic growth. Choi adapted his own chamber music works, even though he seldom adapted other people's music works and also adapted violin concerto in *D* major (Op.61) into the piano concerto version [8]. The romantic period reached the peak of the development of piano adaptation. Bishop and others have left piano adapted works more or less, including famous songs [9]. Among all composers involved in the field of piano adaptation, Liszt's achievements are unmatched. He not only created a large number of piano-adapted repertoires but also brought the technical difficulty and artistic quality in this field to an unprecedented level and also had a far-reaching impact on the subsequent composers' creations.

Under the influence of Voskoboinikov, later composers also continued to explore the road of piano adaptation [10]. By the 20th century, the difficulty of piano adaptation was more challenging, and the path and purpose of adaptation were gradually diversified. Most importantly, the adapted music created for teaching and training has become a new creative direction. Campayo Munoz succeeded Liszt in his prominent position as a leader in the field of piano adaptation. His adaptation achievements are also famous for their large number, wide types, and fine technology [11]. Bugos in addition to the adaptation of Bach's violin and cello works, the adaptation of Chopin etude and waltz is more applied in piano teaching [12]. Park adapted Rimsky–Korsakov's “wild bees flying” as a household name [13]. Mosorsky's “picture exhibition” adapted by Bondarenko is also a common track in today's concert [14]. Pianists Radzetskaya and others also set foot in piano adaptation, adding many wonderful chapters to the piano players' repertoire selection [15]. In today's music environment, piano adaptation has gone deep into every corner of piano learning and performance. From professional piano teaching to popular piano music loved by amateurs, adaptation and creation can be said to be everywhere. Only from the perspective of the scope of professional teaching, the large number of works and repertoires left by predecessors are enough to make us think about the practical significance and teaching value of piano adaptation.

## 3. Methods

The algorithmic compilation, or automated compilation, is a set of rules designed to make a variety of music an organic whole in accordance with certain rules. Algorithm design does not have to be computer [16]. In the classical era, a combination of different music modules was created at random to create a “music cube game” with good results.

### 3.1. Design of the Music Creation Model Based on Hidden Markov

The traditional Markov chain composition method is based on the Markov model. Usually learn a certain amount of music and build a Markov model with note or rhythm as the state space. However, for music, rhythm and melody (pitch fluctuation, i.e., melody) are the two most important elements in music, and they are an inseparable whole. In order to simplify the calculation, only one or a few music elements are usually considered in the algorithm research. However, the current research usually separates the musical elements considered, such as modeling the rhythm and melody separately, which obviously does not meet the needs of music creation. This article will improve this. The hidden Markov model is used to describe the relationship between rhythm and melody of music, and the two are created as related factors, as shown in Figure 3.

HMM is a statistical model of time. It is often used to describe the Markov process that is not clear. Markov procedures are always visible to the observer. The result of global change is all the characteristics of the model. In the HMM, the state is not directly visible, but some changes affecting the state are observed [17]. Because each state has a result of the distribution of possible release codes, the sequence of release signals can present some information about the state temporarily. Therefore, HMM has two result matrixes, the state manifestation matrix and the transmitted disease matrix corresponding to the behavior formed or received when the state changes. An HMM consists of the following five components:

The implied status is

(1) $$\begin{array}{c} X=\left\{x_{1},x_{2},\ldots ,x_{n}\right\}, \end{array}$$

where *n* represents the number of all possible states.

The set of observation symbols is

(2) $$\begin{array}{c} Y=\left\{y_{1},y_{2},\ldots ,y_{m}\right\}, \end{array}$$

where *m* represents the number of possible observation symbols corresponding to each state.

The state transition matrix is

(3) $$\begin{array}{c} A=\left\{a_{ij}\right\}, \end{array}$$

where

(4) $$\begin{array}{c} a_{ij}=p\left(q_{t+1}=x_{j}|q_{t}=x_{i}\right),\;1\leq i,\;j\leq n, \end{array}$$

where *q*_*t*_ represents the state at time *t*.

The emission matrix, the observation probability matrix, is

(5) $$\begin{array}{c} B=\left\{b_{i}\left(k\right)\right\},\;1\leq k\leq m,\;1\leq i\leq n, \end{array}$$

where

(6) $$\begin{array}{c} b_{i}\left(k\right)=p\left(o_{t}=y_{t}|q_{t}=x_{i}\right), \end{array}$$

where *o*_*t*_ represents the observed value in the state of *x*_*i*_ at time *t*.

The initial state is

(7) $$\begin{array}{c} \pi =\left\{\pi_{i}\right\},\;1\leq i\leq n, \end{array}$$

where

(8) $$\begin{array}{c} \pi =p\left(q_{1}=s_{i}\right). \end{array}$$

A simple HMM state transition is shown in Figure 4

Thus, the HMM model can describe the process of transition from a known state to a latent state. In other words, when the sequence analysis *O* = *o*1, *o*2,…, *o*t know when the model is unknown, the probability of the state *Q* = *q*1, *q*2,…, *q*t is choice. This is the decryption problem in HMM. In this sentence, we use the Viterbi algorithm to solve this.

The Viterbi algorithm is a dynamic programming algorithm. It is often used to determine the hidden Markov model to find out the most likely occurrence in state systems that visualize state events as the state is aware of.

Assuming that the state space is *X*, the probability of the initial state *x*_*i*_ is *i*, the state transition probability matrix is A, the emission probability matrix is B, and the observed outputs are *o*1, *o*2,…, *o*t, and the most likely state sequences *q*1, *q*2,…, *q*t that produce the observation results can be recursively obtained by the following formulae:

(9) $$\begin{array}{c} V_{1,x_{i}}=P\left(o_{1}|x_{i}\right)\cdot \pi_{i}, \end{array}$$

(10) $$\begin{array}{c} V_{t,x_{i}}=P\left(o_{t}|x_{i}\right)\cdot \max_{x_{j}\in X}\left(a_{j,k}\cdot V_{t-1,x_{j}}\right). \end{array}$$

Formula (10) is the result of the sequence of states corresponding to the result of the first *t* analysis with the last state *x*_*i*_. The Viterbi method can be obtained by resetting the indicator and alerting the state in a vault (10). In addition, the function Ptr (*x*_*i*_, *t*) is used to refer to *x*_*i*_ for the calculation of *t* > 1 or *t* = 1. Therefore, it is shown as

(11) $$\begin{array}{c} \left\{\begin{array}{c} x_{t}=\arg\max_{x_{j\in X}}\left(V_{t,x_{j}}\right)\\ x_{t-1}=Ptr\left(x_{t},t\right) \end{array}.\right. \end{array}$$

Then, according to the Viterbi algorithm, we can use the known observation state of the system to infer the most likely hidden state.

Rhythm is the skeleton of music. Although the music fluctuates and sounds are elegant, the music can be chaotic if there is no good rhythm in the background. HMM provides a great solution for connecting music and rthyme. In this form, rhyme is considered to be the underlying state of HMM, and music is the latent state in HMM. First, create an assembly and then create a new system of music using the Viterbi algorithm based on this analysis. In previous research by Markov simple concepts, most of them used a form or writing term as a placeholder for states of random processes. For example, the frequency of the next state of each record is considered to be the probability that the current state will move to the next state [18]. This method can only affect the surface structure of the training samples. In order to develop a deeper model, we need to create a more robust Markov chain, which will increase the complexity of the algorithm, and in most cases, the gain will not be lost. In this case, the function extracts information from the data and adds an understanding of the meaning of the music to improve the perception of HMM in the music, as shown in Figures 5–8.

In order to mine the internal structure of music knowledge to the greatest extent on the premise of first-order HMM, this study adopts the learning method of melody element and single note. The melody element construction based on music rules is more similar to the creation mode based on a knowledge base system and music grammar, which will limit the structure of melody elements to a certain extent, and this study has proposed that it is very difficult to build a complete and effective music rule system. In this way, the melody element generation system based on music rules will produce many melody elements that do not meet the requirements. In Karsten Verbeurgt's method, melody elements are extracted based on the dictionary tree query principle, but the length of melody elements is not limited, which will lead to several sections of the learning sample being defined as one melody element at the same time, which sets a great obstacle to the creativity of music creation [19]. Therefore, in this study, the melody element is defined as follows: the music segment that appears more than twice in a piece of music and is between 2 and 5 notes in length is the melody element. The dictionary tree will not be described in detail in this article. We will give an example to introduce how to extract the melody elements in the music clips to be learned according to the dictionary tree search principle. First, we treat all the occurrence positions of each note as a root node and query downward until all branches of a root node have different notes. For example, the code of a piece of music is “ABCABCDE.” The search tree constructed according to this music is shown in Figure 9.

There are three small fragments that have appeared more than twice, ABC, BC, and C. However, the music segment with more than two occurrences and a length between 3 and 5 notes only has ABC. Therefore, according to the definition of melody element in this study, the melody element is ABC.

Through this method, all qualified melody elements in a series of music to be learned can be extracted. When training the transition probability parameter matrix of HMM, melody elements and single notes are fused together to form a state space describing the multilayer structure of music, which makes up for the problem of probability combination between notes that can only describe the surface of music in the first-order Markov [20].

In conclusion, it can be determined that the music you are going to study in the hidden state of HMM has a record and the music is deleted. By definition, the music of music education is a state of observation. The following three parameters need to be defined: state change probability matrix, launch probability matrix, and primary probability matrix. Once we have identified the hidden state of the model, we can calculate the hours of each region in the music segment we need to study. Each state has the ability after the state (warning or travel time), and the frequency of these states is considered to be the resulting matrix for the change of states, as reported in the following equation:

(12) $$\begin{array}{c} a_{ij}=\frac{N\left(q_{j}|q_{i}\right)}{\sum_{k=1}^{n}N\left(q_{k}|q_{i}\right)}, \end{array}$$

where 1 ≤ *j* ≤ *n*, *n* is the number of each state obtained after the current *q*_*i*_ state. N (qk | qi) is the number of next qk states of the current *q*_*i*_ state. For some states, the probability of a change is considered zero unless there are other states. For example, in “ABCABCDE,” state “A” does not jump to “D.” Then, the result of moving from state “A” to state “D” is defined by zero.

The initial probability matrix is the result of the latent state to the visible state. We interpret the data according to the latent state, and the relative time for the data is the state analyst. The probability matrix then counts the total time values of the notes in the music study and their frequency. The formula is the same as the state transition matrix result as shown in the following equation:

(13) $$\begin{array}{c} b_{ij}=\frac{N\left(o_{j}|q_{i}\right)}{\sum_{k=1}^{n}N\left(o_{k}|q_{i}\right)}. \end{array}$$

The first state distribution determines the initial state of the model. This information counts the location and number of first points of all text in each music section to be studied. The first result of the recording is given in the following equation.

(14) $$\begin{array}{c} \pi_{i}=\frac{N\left(q_{i}\right)+1/\text{index}\left(q_{i,1}\right)}{\sum_{j=1}^{n}N\left(q_{j}\right)+\sum_{j=1}^{n}1/\text{index}\left(q_{j,1}\right)}. \end{array}$$

Here, 1 ≤*i* ≤ *n*, *n* is the size of the state model, and *N* (*q*_*i*_) is the number of events of the state *q*_*i*_ in the training model. Imolex (*q*_*i*_) is the state function that first appeared during the training sample package. The initial probability of a given state is proportional not only to its frequency in the sample set but also to its position in a given text. It can reflect the rule of this state in this sample set.

Because the surface structure of the music is important, it often indicates time and security. Thus, these data initiate the first Markov chain decision of the state analysis of the model [21]. The time interval in the set structure is taken to be the local state, and the frequency of the resulting states is calculated from the occurrence of the initial distribution and the transition state matrix (12). To simplify the algorithm, the length of the system type created by the model is limited to 50. The flow diagram of the composite system as HMM is shown in Figure 10.

### 3.2. Interactive Genetic Algorithm Optimization Model

Theoretically, the HMM-based design algorithm proposed in this article can produce music similar to training models, but music is a commercial product that has good wishes. Different people may have different opinions about songs of the same genre. Therefore, it is important to consider how the music composing algorithm can create a sound that meets the needs of the users [22]. To solve this problem, this sentence uses an interactive genetic algorithm. On the other hand, the crossover operator of the genetic algorithm retains the excellent performance in the music production equipment, and the exchange operator can not only learn from the performance but also changes the music like the creative attitude of the composer who gives it all, playing with their inspiration in acting. On the other hand, an interactive genetic algorithm uses measurement tools, which allow the evolution of music to suit the user's needs and thus to the user's needs. Music encoding uses MIDI encoding numbers. Considering the training examples selected in this article, atherosclerosis coding is limited to thirty-six sheets for all studies [23]. The time of the entire map is defined in the first unit, and the audio encoding is [1/32, 1/16, 1/8, 1/4, 1/2, 1]. The music is finally encoded into the matrix, as reported in the following equation:

(15) $$\begin{array}{c} \mathrm{chrom}=\left[\begin{array}{cccc} 58 & 60 & 61 & 62\\ 0.5 & 0.25 & 0.25 & 0.5 \end{array}\right]. \end{array}$$

The pitch of the first behavior and the rhythm value of the second behavior.

Select operator and operator crossover as a roulette option and multiple themes crossover. The following three exchange rates are used by exchange staff:

(1) A segment of pitch in a chromosome increases or decreases *n* steps at the same time, and the variation range of *n* is set as [1, 2, 3], as shown in the following formula:
  (16) $$\begin{array}{c} chrom\_\text{mu}=\text{chrom}\pm \left[\begin{array}{cccc} n & n & n & n\\ 0 & 0 & 0 & 0 \end{array}\right]. \end{array}$$
(2) A rhythm in a chromosome increases or decreases K beats at the same time, and the value range of K is [0.25, 1, 1.5, 2], as shown in the following formula:
  (17) $$\begin{array}{c} \text{chrom}=\text{chrom}\pm \left[\begin{array}{cccc} 0 & 0 & 0 & 0\\ k & k & k & k \end{array}\right]. \end{array}$$
(3) Single point random mutation:

When there is a change, if the notice or value match exceeds the limit, it will randomly move to the state in its respective state.

This phrase is used to measure the book to provide exercise value to the music and to be the leader of the improvement. To reduce the hearing of users during the evolution of the algorithm, the physical value of a person is determined by weight of book analysis and similar according to the morphological characteristics of the music, as shown in the following equation.

(18) $$\begin{array}{c} Fit\left(i\right)=w\cdot H\left(i\right)+\left(1-w\right)\cdot S\left(i\right). \end{array}$$

Among them, *H* (*i*) and *S* (*i*) are the normalized manual evaluation value and similarity based on music morphological features, respectively, and *w* is the weight of connecting the two parts of fitness. The value rule is shown in the following formula:

(19) $$\begin{array}{c} w=\left\{\begin{array}{cc} 1, & n=\lambda \cdot k-\frac{k\cdot \left(k-1\right)}{2}\cdot \beta ,n>100,\lambda -k\cdot \beta \geq 0,\\ 0, & \text{else,} \end{array}\right. \end{array}$$

where *n* is the evolutionary algebra, *kϵ N*, *N* is a natural number, and *β* and *λ* are the positive integers. In this study, 20 and 4 are taken, respectively. This can ensure that the artificial evaluation can completely dominate the evolution direction with the evolution algebra.

Similar pitch and rhythm can express similar hearing. The fitness when *w* is 1 is given by the user. When *w* is 0, using the morphological characteristics of the optimal individual to measure the advantages and disadvantages of population evolution can also achieve the purpose of guiding evolution in the direction of user needs [24]. In this study, the morphological characteristics of note sequence are symbolized, and rising, stationary, and falling are mapped as [1, 0, −1], respectively. Then, the fitness function of the individual is calculated by using the similarity of morphological features, as shown in the following formula:

(20) $$\begin{array}{c} S\left(i\right)=\sum_{j=1}^{l-1}\sqrt{{\left(SPop\left(i,j\right)-Sbest\left(j\right)\right)}^{2}}, \end{array}$$

where *l* is the length of the individual, and SPop and Sbest are the symbolized population and the best individual, respectively.

Through fitness formula (18), the termination condition of the algorithm is to reach the maximum evolutionary algebra or user satisfaction. To sum up, the flowchart of the composition algorithm based on HMM and IGA proposed in this study is shown in Figure 11.

## 4. Experimental Results and Discussion

This article describes the simulation method based on MATLAB. Example training: classical piano performance. The parameters algorithm is developed as follows: The length of the design work is 50 notes. The length of the text is obtained from the dictionary looking for trees [2,5]. The magnitude of the IGA population is 10, the maximum evolutionary algebra is 50, the crossover probability is 0.8, and the correlation probability is 0.2. Equation (19) *λ* is 20, *β* is 4, and formula (16) has a range of N oscillations [1–3]. The average in equation (19) is 4 because of 20, so the simulation yields 4 false positives. Each column represents the physical values of the four false tests in a simulation. With the exception of four simulations, it can be seen that the algorithm can achieve sufficient results, as shown in Figures 12–15.

Compared to Markov's compositional algorithm, this algorithm not only considers the possibility of isolating notes and rhythms but also combines notes and rhythms, elements of the movement, and the mapping between rhythms with elements of the movement. The creations are more coherent, adaptive, and have a sense of rhythm. Compared to other popular neural network-based algorithms, this algorithm has advantages such as fast learning speed, small samples, and human-computer interactions [25], as shown in Figure 16.

Piano adaptation is a link that cannot be ignored in the field of piano art. This form of music creation integrates social change, class change, and artistic trends. Digging deeply into the theory, the piano adaptation reflects a kind of extreme pursuit that evolved from the development of Western classical music in the 19th century; while observing from the practical application, this phenomenon is related to the popularization aesthetics of mass entertainment. Based on its remarkable achievements in the history of music development and its application in today's performance and teaching, the importance of piano adaptation is self-evident. To sum up, piano adaptation has played a positive role in the development of piano art. Although its esthetic taste has two-sided characteristics, it cannot erase the historical and artistic value of such works. The development path of Chinese piano adaptation is different from that of the West, but they all provide wonderful artistic chapters for piano players. The selection of excellent piano adaptation is helpful to improve the player's vision and skills, to enrich artistic expression, and has a practical significance in teaching and performance practice.

## 5. Conclusion

This line presents an interesting way to research to become our leader in psychiatry and creativity in various fields of music. The simulation results show that the new computer-based functionality based on the hidden Markov model and the interactive genetic algorithms mentioned in this article can be used to create cohesive working groups, such as model training and guiding the evolution of development. The next step is to develop an algorithm tailored to the needs of the users and ultimately to create activities that satisfy the customer. The algorithm is less complicated and requires less examples of training. I believe that in the age of information and knowledge of the future, we will explore our mental performance of control and creativity of ourselves using Markov's secret model and interactive genetic algorithms in a variety of music environments.

## Figures and Tables

**Figure 1:** Summary of theory, technology, and practice.

**Figure 2:** Multicultural music flowchart.

**Figure 3:** Creation flowchart.

**Figure 4:** HMM state transition diagram.

**Figure 5:** Comparison of loss function values of different LSTM units.

**Figure 6:** Comparison of loss function values of different LSTM layers.

**Figure 7:** Comparison of loss function values of different scales.

**Figure 8:** Comparison of loss function values of different track numbers.

**Figure 9:** Melody meta-search tree constructed according to “ABCABCDE.”

**Figure 10:** Flowchart of the composition algorithm based on HMM.

**Figure 11:** Computer composition algorithm based on HMM-IGA.

**Figure 12:** The number of iterations is 200.

**Figure 13:** The number of iterations is 400.

**Figure 14:** The number of iterations is 600.

**Figure 15:** The number of iterations is 1000.

**Figure 16:** Note category frequency diagram.

## Data Availability

The dataset used to support the findings of this study is available from the corresponding author upon request.
